This article has been retracted.

# The Value of Artificial Intelligence Film Reading System Based on Deep Learning in the Diagnosis of Non-Small-Cell Lung Cancer and the Significance of Efficacy Monitoring: A Retrospective, Clinical, Nonrandomized, Controlled Study

**DOI:** 10.1155/2022/2864170

**Published:** 2022-03-22

**Authors:** Yunbing Chen, Xin Tian, Kai Fan, Yanni Zheng, Nannan Tian, Ka Fan

**Affiliations:** Department of Computerized Tomography, Jincheng People's Hospital (Jincheng Hospital Affiliated to Changzhi Medical College), No. 456 Wenchang East Street, Jincheng, 048026 Shanxi, China

## Abstract

**Objective:**

To explore the value of artificial intelligence (AI) film reading system based on deep learning in the diagnosis of non-small-cell lung cancer (NSCLC) and the significance of curative effect monitoring.

**Methods:**

We retrospectively selected 104 suspected NSCLC cases from the self-built chest CT pulmonary nodule database in our hospital, and all of them were confirmed by pathological examination. The lung CT images of the selected patients were introduced into the AI reading system of pulmonary nodules, and the recording software automatically identified the nodules, and the results were compared with the results of the original image report. The nodules detected by the AI software and film readers were evaluated by two chest experts and recorded their size and characteristics. Comparison of calculation sensitivity, false positive rate evaluation of the NSCLC software, and physician's efficiency of nodule detection whether there was a significant difference between the two groups.

**Results:**

The sensitivity, specificity, accuracy, positive predictive rate, and false positive rate of NSCLC diagnosed by radiologists were 72.94% (62/85), 92.06% (58/63), 81.08% (62+58/148), 92.53% (62/67), and 7.93% (5/63), respectively. The sensitivity, specificity, accuracy, positive prediction rate, and false positive rate of AI film reading system in the diagnosis of NSCLC were 94.12% (80/85), 77.77% (49/63), 87.161% (80 + 49/148), 85.11% (80/94), and 22.22% (14/63), respectively. Compared with radiologists, the sensitivity and false positive rate of artificial intelligence film reading system in the diagnosis of NSCLC were higher (*P* < 0.05). The sensitivity, specificity, accuracy, positive prediction rate, and negative prediction rate of artificial intelligence film reading system in evaluating the efficacy of patients with NSCLC were 87.50% (63/72), 69.23% (9/13), 84.70% (63 + 9)/85, 94.02% (63/67), and 50% (9/18), respectively.

**Conclusion:**

The AI film reading system based on deep learning has higher sensitivity for the diagnosis of NSCLC than radiologists and can be used as an auxiliary detection tool for doctors to screen for NSCLC, but its false positive rate is relatively high. Attention should be paid to identification. Meanwhile, the AI film reading system based on deep learning also has a certain guiding significance for the diagnosis and treatment monitoring of NSCLC.

## 1. Introduction

Lung cancer is the highest incidence of malignant tumor in the world. In recent years, the morbidity and mortality have increased year by year, and it has become the leading cause of tumor-related death [1, 2]. About 80% of lung cancer patients are non-small-cell lung cancer (NSCLC), of which advanced patients account for 40% of the total number of NSCLC patients. The mortality rate in the same period increased by 9% over 2007, accounting for 28.6% of tumor-related deaths [3, 4]. According to the statistics of the National Cancer Prevention and Research Office of the Ministry of Health, the estimated and predicted deaths of lung cancer in China are increasing year by year. The estimated number of lung cancer deaths in 2005 is more than double that in 1991 [5]. In recent years, China's natural population growth, population aging process intensified, rural urbanization, and urban industrialization process are also accelerating; the number of smokers in China is also increasing year by year, and the above reasons are the main factors for the linear increase in the incidence of lung cancer in China in recent years. For a long time, lung cancer ranks first in the incidence and mortality of malignant tumors in China [6–8]. It has become an important public health problem that seriously affects the health of Chinese residents. NSCLC has a high degree of malignancy, which usually occurs in the elderly, and the prognosis of the patients is generally poor.

Early lung cancer lacks typical symptoms and generally comes to see a doctor when the patient's condition progresses and secondary symptoms appear [9]. NSCLC can be characterized by irritating dry cough, occasionally with blood in sputum; when the tumor grows rapidly or involves the recurrent laryngeal nerve, patients often go to see a doctor because of hoarseness; when they invade the visceral pleura, pleural effusion can be accompanied by pleuria [10]. Patients often come to see a doctor because of chest stifling and wheezing. At this time, the degree of tumor invasion is deep, the best operation time has been lost, and the prognosis is poor [9, 10]. Some studies have suggested that early detection and early treatment of tumors can increase the five-year survival rate of patients from 14% to 49% [11]. Therefore, early diagnosis of NSCLC and timely adoption of the correct treatment plan are of vital clinical significance to improve the prognosis of patients and improve the quality of life.

The diagnosis of lung cancer is mainly divided into two parts, including localization diagnosis and qualitative diagnosis. Qualitative diagnosis is the key to the accurate diagnosis of lung cancer, which is directly related to the follow-up treatment of patients. The traditional qualitative diagnosis includes bronchoscopic tissue biopsy, mediastinal lymph node biopsy, pleural effusion exfoliative cytology, percutaneous lung biopsy, and surgical pathology [12]. These procedures have certain risks and cause trauma to patients, and even complications such as pneumothorax, hemothorax, and pleural reaction occur in improper operation.

Till now, imaging examination has great advantages in the diagnosis, staging, and grading of lung cancer and has gradually become an important way to evaluate lung cancer. At present, chest X-ray and computed tomography (CT) are commonly used in clinical work, followed by nuclear magnetic resonance imaging (MRl) and positron emission computed tomography (PET/CT).

Chest X-ray is the most basic examination method, which is often used as a screening method for lung cancer and other lung diseases. However, due to the low density resolution and overlapping images of various tissues and organs, it is easy to induce missed diagnosis and misdiagnosis of early lung cancer. Patients miss a good opportunity for treatment, so there are some limitations [13]. The appearance of chest CT imaging technology makes up for the problem of image overlap caused by chest film and improves the image density resolution. At present, the most widely used multislice spiral CT further improves the scanning speed and intelligently processes the image through postprocessing techniques, such as multiplane reconstruction, maximum/minimum density projection, surface shaded display and volume rendering, and virtual endoscopy, to more accurately analyze the basic imaging features of the lesions. It is beneficial to the localization and qualitative diagnosis of lesions and has become the most commonly used imaging examination method for the diagnosis of lung cancer [14]. However, CT still has some defects, such as high radiation dose; it is difficult to distinguish similar inflammation and tumor lesions, and the complex structure and components of lung cancer cannot be evaluated only by measuring CT values. The greatest advantage of magnetic resonance imaging is that it has high resolution for soft tissue. A variety of sequences are conducive to the evaluation of the internal components of the lesions and play a central role in the qualitative, differential diagnosis, and metastatic lymph node evaluation of pulmonary space occupying. However, the application of MRI in chest imaging is relatively less, mainly due to the high price and long examination time, and the image quality is unstable [15]. PET-CT can combine functional metabolic imaging with CT imaging. At present, it is mainly used to locate the focus and evaluate the whole body metastatic foci. However, due to the limitation of the use of drugs, the examination is very expensive, and the radiation dose is high, so PET-CT has not been widely used in clinical work [16].

In recent years, big data and artificial intelligence (AI) are booming in the medical field. AI based on deep learning is widely used in image detection, pathological diagnosis, diagnosis and treatment planning, and survival prediction. Based on the basic data of disease spectrum and the deep learning model based on convolution neural network (CNN), a computer aided diagnosis (CAD) system is established. The application of AI technology in the detection of pulmonary nodules in chest CT images is a hot topic in the current research. This study discussed the value of AI film reading system based on deep learning in the diagnosis of NSCLC and the significance of curative effect monitoring. The report is as follows.

### 1.1. Patients and Methods

#### 1.1.1. Objective of Study

The images of 104 cases of suspected lung cancer in the self-built chest CT pulmonary nodule database of our hospital were selected retrospectively. The criteria were as follows: (1) the patient with at least 1 noncalcified nodule, (2) the patient who had thin chest CT images (slice thickness ≤ 1.25 mm), and (3) the patient was confirmed by pathological examination with the nature of pulmonary nodules. (4) Images with diffuse metastasis, interstitial lung disease, extensive scarring, pneumonia, fibrosis, pulmonary edema, and severe motion artifacts were excluded.

#### 1.1.2. CT Scanning Technology

All examinations were performed by 16-row (Siemens Emotion16) 64-row (Toshiba Aquillion 64) spiral CT machines. The scanning range is from the entrance of the chest to the base of the lung. The patient takes a breath and then holds his breath to complete the whole lung scan. Scanning mode: was butterfly scan; tube voltage was 120 kV or 140 kV tube current: was 200 mA-340 mA; pitch: 1.37; slice thickness: was 5.0 mm; image matrix: was 512 × 512; visual field (field of view (FOV)): 360 mm. was The axial images of 1.25 mm slice thickness were reconstructed using the standard algorithm.

#### 1.1.3. Diagnostic Method of Pulmonary Nodules

The radiologists, two middle-aged radiologists (6 years and 7 years of service, respectively), were used to determine the nodular nature of the CT findings of 104 patients. The different results were determined by the joint discussion of two radiologists.

For AI film reading system, the AI film reading software (Deepwise Healthcare, V1.3.0.1) based on deep learning model is provided by Shenrui Medical Co., Ltd., which transmits the raw data of chest CT to the workstation, and the software system automatically identifies and marks pulmonary nodules in batches. Convolution neural network (CNN) is a deep learning algorithm which is often used in the field of image recognition and processing, such as face recognition and other related fields. The main components of CNN are convolution layer, pooled layer, and fully connected layer (FC). The convolution layer uses a specific size of convolution to check image convolution so as to learn and extract abstract and deep features. The pooling layer is often placed after the convolution layer, and the main function is to compress and reduce the dimension of the extracted features, so as to reduce the amount of operational data. The fully connected layer mainly maps the final features to the output layer. After the successful processing of the workstation, according to the recognition of pulmonary nodules in the chest CT images on the display interface of the workstation, the detection results of pulmonary nodules in the depth learning model were recorded.

#### 1.1.4. Nodule Standard Identification

Pathological examination was used as the gold standard for the diagnosis of NSCLC, and the size, location, and density of each noncalcified nodule were recorded. The size of nodules was divided into three groups: <5 mm, 5 mm-10 mm, and >10 mm. The location of the nodules was divided into four groups: connected to the pleura, peripheral nodules (within the pleural 2 cm, but not connected to the pleura), hilar nodules (within the hilar 2 cm), and central nodules (located between the peripheral and hilar nodules). According to the nodule density, the patients were divided into three groups: solid nodule, partial solid nodule, and ground glass density nodule. Ground glass density nodules are defined as fuzzy nodules in the lung, which are slightly denser than lung tissue, and do not cover lung texture structures such as bronchi and blood vessels, while some solid nodules are defined as containing both ground glass density components and solid soft tissue density components.

#### 1.1.5. Treatment Methods

Patients with diagnosed NSCLC were given routine treatment, thoracoscopic lobectomy/segmental lobectomy was performed after excluding surgical contraindications, and adjuvant radiotherapy and chemotherapy were given during the perioperative period. After treatment, the outpatients were followed up for 1 year, once every month.

#### 1.1.6. Evaluation Method of Curative Effect

After the patients with diagnosed non-small-cell lung cancer received systematic and regular treatment, the therapeutic effect was evaluated by 2 chest imaging experts and 2 thoracic surgery experts according to the patients' clinical manifestations, laboratory indexes, and imaging examination as the gold standard. The therapeutic effect is divided into effective and ineffective.

#### 1.1.7. Statistical Analysis

The SPSS 22.0 statistical software was used for data entry, collation, and statistical analysis. The sensitivity and false positive rate of artificial intelligence film reading system and imaging physician in detecting NSCLC were calculated, respectively. Chi-square test was used to compare the ability of artificial intelligence film reading system and imaging physician in the diagnosis of non-small-cell lung cancer. The difference was statistically significant (*P* < 0.05).

## 2. Results

### 2.1. Results of Pathological Examination of Pulmonary Nodules

The results of pathological examination in 104 patients with pulmonary nodules showed that a total of 148 noncalcified nodules were detected. The size, location, and density distribution of noncalcified nodules are as follows. All the data are presented in Table 1.

### 2.2. Results of Radiologist's Diagnosis of NSCLC

The sensitivity of radiologists in the diagnosis of NSCLC is 72.94% (62/85), the specificity is 92.06% (58/63), the accuracy is 81.08% ((62 + 58)/148), the positive predictive rate is 92.53% (62/67), and the false positive rate is 7.93% (5/63). All the data are presented in Table 2.

### 2.3. Results of Artificial Intelligence Film Reading System in the Diagnosis of NSCLC

The sensitivity of artificial intelligence film reading system in the diagnosis of NSCLC is 94.12% (80/85), the specificity is 77.77% (49/63), the accuracy is 87.161% ((80 + 49)/148), the positive predictive rate is 85.11% (80/94), and the false positive rate is 22.22% (14/63). All the data are presented in Table 3.

### 2.4. Comparison of the Efficacy of Radiologist and Artificial Intelligence Film Reading System in the Diagnosis of NSCLC

Compared with radiologists, the sensitivity and false positive rate of artificial intelligence film reading system in the diagnosis of NSCLC were higher, and the difference was statistically significant (*P* < 0.05). All the data are presented in Table 4.

### 2.5. Evaluation of Curative Effect in Patients with NSCLC by Artificial Intelligence Film Reading System

The sensitivity, specificity, accuracy, positive prediction rate, and negative prediction rate of artificial intelligence film reading system in evaluating the efficacy of patients with NSCLC were 87.50% (63/72), 69.23% (9/13), 84.70% ((63 + 9)/85), 94.02% (63/67), and 50% (9/18), respectively. All the data are presented in Table 5.

### 2.6. Misdiagnosis of NSCLC Diagnosed by Radiologist and Artificial Intelligence Film Reading System

Figure 1(a) shows the imaging results of a 56-year-old male patient, the artificial intelligence film reading system was diagnosed as suspected lung cancer in the left upper lung, and the radiologist reported that the left upper lung was space occupying considering granulomatous inflammation. Later, it was diagnosed as granulomatous inflammation of the left upper lung by puncture pathology, which was inclined to pulmonary tuberculosis. Figure 1(b) shows the focus shrinking and absorbing after 2 months of antituberculosis treatment. Figure 1(c) shows the imaging results of a 61-year-old female patient. The artificial intelligence film reading system was diagnosed as suspected lung cancer in the right upper lung, and pneumonia was considered for the right upper lung mass as reported by the radiologist. It was diagnosed as right upper lung organic pneumonia by puncture pathology. Figure 1(d) shows that the focus was basically absorbed after 3 months of anti-infective treatment.

## 3. Discussion

According to the global cancer epidemiological statistics released by the American Cancer Society in 2018, there are 2.1 million new cases of lung cancer and 1.8 million deaths worldwide, accounting for 11.6% of the total number of cancer cases and 18.4% of the total cancer deaths [18]. In recent years, although the screening technology of lung cancer has been making continuous progress, because most of the early lung cancer has no obvious symptoms and signs, when there are typical symptoms such as hemoptysis and chest pain, the course of the disease has entered the middle and late stage, which is easy to relapse and metastasis. The therapeutic effect is not ideal [19]. According to reports, patients with NSCLC who are locally advanced diseases at the time of diagnosis account for about 60% of all patients [20]. At present, the prognosis of these patients is poor, with a 5-year survival rate of 15% in locally advanced non-small-cell lung cancer (LA-NSCLC) and only 5% in advanced NSCLC [21]. Due to the lack of typical clinical manifestations in the early stage of lung cancer, the sensitivity and specificity of early screening methods of lung cancer, such as chest X-ray, sputum cytology, and serum oncology, are not high, and the role in early screening is limited. Pulmonary nodule is the most important early imaging manifestation of lung cancer [22]. CT significantly increased the detection rate of pulmonary nodules. Thin-slice CT technology is more helpful to detect smaller pulmonary nodules, but thin-layer CT significantly increases the number of chest CT imaging and the reading quantity of radiologists. Radiologists may miss diagnosis and misdiagnosis due to inexperience and fatigue.

In the 1970s, the computer-aided detection and diagnosis (CAD) system came into being. The application of CAD in the medical field can be traced back to a literature on automatic detection of lesions by computer in Radiology in 1967, but due to the limitation of computer performance at that time, it could not achieve good experimental results; until 1985, Kunio Takai of Chicago University first puts forward the basic concept of CAD [23]. CAD refers to the software system that uses computer to assist in the detection and diagnosis of various diseases, including computer-aided detection system (CADe) and computer-aided diagnosis system (CADx). In the detection of chest CT pulmonary nodules, the CADe system based on chest CT examination has attracted wide attention. CADe can initially screen a large number of chest CT images and mark suspicious lesions, so as to help radiologists to make secondary discrimination, so as to reduce the workload and improve the efficiency of screening. Traditional CADe systems usually consist of two main stages: (1) selection of candidate nodules (that is, differential nodules) and (2) removal of false positive nodules (FPN) while preserving true positive nodules (TPN) (that is, candidate nodules are divided into nodules or nonnodules). FPN is often excluded in the second stage of classification. A lot of work has been done to extract various specific features such as morphology (such as size and roundness), gray level (such as histogram features), or texture from segmented or unsegmented images and input them into support vector machines (SVM), decision trees (DecisionTree), and artificial neural networks (ANN) [24, 25]. There are many literatures to summarize the traditional CADe system. Wormanns et al. studied the traditional CADe system, and the sensitivity of radiologists and CADe were 90% and 24%, respectively, especially for nodules connected to the pleura, but higher sensitivity to nodules in the central area that were easily misdiagnosed as vascular structures by radiologists [26, 27]. Some studies have also shown that the sensitivity of traditional CADe system to ground glass density nodules is low [28]. The traditional CADe system has shown good effectiveness in some aspects of pulmonary nodule detection, but the traditional CADe system only detects pulmonary nodules according to local characteristics from a statistical point of view, which cannot meet the needs of high sensitivity and low false positive in pulmonary nodule detection [27].

In recent years, with the application of big data and the improvement of computer computing ability, deep learning algorithm has been developed rapidly. Deep learning technology can effectively complete the tasks of image detection, recognition, and classification, so the deep learning technology in the field of imaging may help radiologists to complete a variety of diagnosis tasks [28]. The detection of pulmonary nodules using artificial intelligence (AI) algorithm is an important part of the medical field of AI [29]. Different from the traditional machine learning methods that need to extract artificial design features, deep learning can learn abstract and deep image features directly from the original image data [30]. Therefore, deep learning technique has been widely used in CADe of thoracic CT pulmonary nodules. Among them, convolution neural network (CNN) is a deep learning algorithm with multilayer prefeedback structure, which can be used to learn multiple features by using supervised learning and/or unsupervised learning methods. CNN has achieved great success in image processing and has been introduced into the field of medical images. There have been many studies on the application of CNN to the CADe system of pulmonary nodules.

AI, a branch of computer science, is a new technological science that studies theories and application systems used to imitate and expand human intelligence. With the large-scale application of big data, the significant improvement of computer computing power, and the obvious progress of machine learning algorithms, a great breakthrough has been made in the development and application of AI [31]. AI can obtain all kinds of information from the image which is easy to be ignored and/or cannot be extracted by the naked eye, so as to improve the diagnostic efficiency of the image. Using AI technology to detect pulmonary nodules is a key field in the development of artificial intelligence medical industry. Machine learning (ML) is a branch of AI. Deep learning is a kind of machine learning, and it is also the most important branch [31]. This study surveyed the value of AI film reading system based on deep learning in the diagnosis of NSCLC and the significance of curative effect monitoring.

The results of our study showed that the sensitivity, specificity, accuracy, positive predictive rate, and false positive rate of NSCLC diagnosed by radiologists were 72.94% (62/85), 92.06% (58/63), 81.08% (62 + 58/148), 92.53% (62/67), and 7.93% (5/63), respectively. The sensitivity, specificity, accuracy, positive prediction rate, and false positive rate of AI film reading system in the diagnosis of NSCLC were 94.12% (80/85), 77.77% (49/63), 87.161% (80 + 49/148), 85.11% (80/94), and 22.22% (14/63), respectively. Compared with radiologists, the sensitivity and false positive rate of artificial intelligence film reading system in the diagnosis of NSCLC were higher (*P* < 0.05). The results showed that the sensitivity of radiologists in detecting pulmonary nodules was significantly lower than that of the AI software. However, most of the false negative nodules are micronodules with diameter less than 5 mm, and the malignant probability of such nodules is often low. The main reasons include that the radiologist's detection results in this study are based on archived imaging reports, but for some micronodules, small nodules, and/or special nodules, the physician may think that the detection of pulmonary nodules is of little significance, such as interlobar fissure nodules, which may be an important factor in the missed diagnosis of pulmonary nodules. Due to heavy workload, fatigue, and/or lack of experience, it may be unavoidable for radiologists to make a diagnosis only by relying on horizontal axial images or even with reference to thick images, while small nodules are similar to the axial projection of vascular cross-sections, which is prone to result in missed diagnosis or misdiagnosis, which may be another important reason for missed diagnosis and misdiagnosis of pulmonary nodules. AI can indeed help radiologists in nodule detection, but from the point of view of clinical application, the clinical significance of this kind of nodules is still debatable. Further clinical intervention of such nodules completely according to the results of AI will increase medical burden and occupy medical resources. Therefore, further analysis will be carried out, in order to judge whether clinical treatment is needed or not that doctors and AI need to face.

On the other hand, the false positive rate of the AI software was significantly higher than that of radiologists. The cause of false positive may be related to the extremely low threshold for detecting nodule size set by artificial intelligence software. After we removed the false positive nodules smaller than 5 mm, the false positive rate was reduced by about 2 × 3. The false positive rate of radiologists in this study is very low; the fundamental reason is that radiologists have more experience in judging false positive nodules than the AI software, while AI focuses more on the learning of positive nodules at the present stage. There is still a lack of learning for false positive nodules. Judging from the misdiagnosis results of AI, it seems that the software cannot effectively distinguish nonnodular structures with similar nodular appearance and/or localized normal or abnormal swollen internal and external structures with significant density differences from surrounding tissues. Figure 1 of the results of this study can be shown laterally. In this study, we found that the AI software performed poorly in patients with diffuse interstitial lung disease, extensive scar formation, pneumonia, fibrosis, edema, and other lung diseases, and the false positive rate was very high, so these cases were excluded. For the cases with local interstitial lesions, pneumonia, fibrosis, and scar formation, there is also the problem of high false positive rate detected by AI, and radiologists have rich clinical experience to distinguish these lesions easily. This may be one of the reasons for the high false positive rate of AI. In clinical practice, patients with malignant pulmonary nodules are often accompanied by these manifestations, so the diversity of training sets should be increased to improve the universality of human AI and achieve a satisfactory false positive rate. Higher false positive results may lead to patients' excessive anxiety and unnecessary intervention, which may cause potential damage and may also render imaging doctors to spend more time to distinguish, and it is also easy to cause misdiagnosis. Therefore, the AI cannot be used as an independent technology in daily work. However, with the improvement of the operation speed of the deep learning model, the continuous accumulation of experience, and the continuous iteration of the model, the diagnostic sensitivity and accuracy can also be improved.

At present, the evaluation of the curative effect and the prediction of prognosis after tumor chemotherapy are mainly based on the morphological indexes—the change of tumor diameter and the change of tumor volume. This study found that the AI film reading system based on deep learning also has a certain guiding significance for the diagnosis and treatment monitoring of NSCLC. The sensitivity, specificity, accuracy, positive prediction rate, and negative prediction rate of AI film reading system in evaluating the efficacy of patients with NSCLC were 87.50% (63/72), 69.23% (9/13), 84.70% ((63 + 9)/85), 94.02% (63/67), and 50% (9/18), respectively. The change of tumor volume is an important evaluation index in the monitoring and follow-up of tumor treatment. Concomitantly, if the imaging image is incomplete and the image quality changes physically over time, it is necessary to compare the images of different periods and view multiple pictures, as well as diagnostic differences among different imaging experts, so that the accuracy of the diagnosis is significantly reduced. AI based on deep learning algorithm can make up for these shortcomings. AI can automatically register and process the multitemporal images of MRI/CT at different time nodes before and after treatment, learn and extract the corresponding features of tumor texture and heterogeneity, fuse the quantitative features of multimodal imaging, including PET-CT and MRI, accurately identify the areas of tumor changes, and give the hotspot map of tumor internal changes. Furthermore, it assists the clinical experts to judge the curative effect of the treatment and greatly reduces the workload of the imaging experts simultaneously.

However, the limitation of this study is that the selection criteria of the number of cases in the data set is based on retrospective case selection, all the cases are found by doctors, and the missed cases in clinic cannot be obtained through retrospective case selection, so there is a certain selective bias.

Taken together, the AI film reading system based on deep learning has higher sensitivity for the diagnosis of NSCLC than radiologists and can be used as an auxiliary detection tool for screening NSCLC, but its false positive rate is relatively high, so attention should be paid to identification. Concomitantly, the AI film reading system based on deep learning also has a certain guiding significance for the diagnosis and treatment monitoring of NSCLC.

## Figures and Tables

**Figure 1:** Misdiagnosis of NSCLC diagnosed by radiologist and artificial intelligence film reading system.

**Table 1:** Univariate analysis in patients with NSCLC (*n* (%)).

Noncalcified nodule	Number (*n* = 148)	Constituent ratio (%)
Size		
<5 mm	72	48.65
5 mm-10 mm	51	34.46
>10 mm	25	16.89
Position		
Connected to the pleura	31	20.95
Peripheral nodule	79	53.38
Hilar nodule	29	19.59
Central nodule	9	6.08
Density		
Solid nodule	86	58.11
Partial solid nodule	12	8.11
Ground glass density nodules	50	33.78

**Table 2:** Results of diagnosis of NSCLC by radiologists (example).

Radiologist	Results of pathological examination		Total
	Positive	Negative	
Positive	62	5	67
Negative	23	58	81
Total	85	63	148

**Table 3:** Results of artificial intelligence film reading software in the diagnosis of NSCLC (example).

Artificial intelligence film reading system	Results of pathological examination		Total
	Positive	Negative	
Positive	80	14	94
Negative	5	49	54
Total	85	63	148

**Table 4:** Comparison of the efficacy of radiologists and artificial intelligence film reading system in the diagnosis of NSCLC.

Diagnostic method	Sensitivity	Specificity	Accuracy rate	Positive predictive value	False positive rate
Radiologist	72.94%	92.06%	81.08%	92.53%	7.93%
Artificial intelligence film reading system	94.12%	77.77%	87.16%	85.11%	22.22%
*χ* ^2^	13.853	3.136	2.028	2.075	5.020
*P*	<0.001	0.076	0.152	0.149	0.025

**Table 5:** Artificial intelligence film reading system to evaluate the curative effect of patients with NSCLC (example).

Artificial intelligence film reading system	Gold standard		Total
	Effective	Invalid	
Effective	63	4	67
Invalid	9	9	18
Total	72	13	85

## Data Availability

The data used to support the findings of this study are available from the corresponding author upon request.
